# Syncytiotrophoblast Microvesicles Released from Pre-Eclampsia Placentae Exhibit Increased Tissue Factor Activity

**DOI:** 10.1371/journal.pone.0026313

**Published:** 2011-10-14

**Authors:** Chris Gardiner, Dionne S. Tannetta, Carol A. Simms, Paul Harrison, Christopher W. G. Redman, Ian L. Sargent

**Affiliations:** 1 Nuffield Department of Obstetrics and Gynaecology, University of Oxford, Level 3, Women's Centre, John Radcliffe Hospital, Oxford, United Kingdom; 2 Oxford Haemophilia & Thrombosis Centre, Churchill Hospital, Oxford, United Kingdom; Brigham and Women's Hospital, United States of America

## Abstract

**Background:**

Pre-eclampsia is a complication of pregnancy associated with activation of coagulation. It is caused by the placenta, which sheds increased amounts of syncytiotrophoblast microvesicles (STBM) into the maternal circulation. We hypothesized that STBM could contribute to the haemostatic activation observed in pre-eclampsia.

**Methodology/Principal Findings:**

STBM were collected by perfusion of the maternal side of placentae from healthy pregnant women and women with pre-eclampsia at caesarean section. Calibrated automated thrombography was used to assess thrombin generation triggered by STBM-borne tissue factor in platelet poor plasma (PPP). No thrombin was detected in PPP alone but the addition of STBM initiated thrombin generation in 14/16 cases. Pre-eclampsia STBM significantly shortened the lag time (LagT, P = 0.01) and time to peak thrombin generation (TTP, P = 0.005) when compared to normal STBM. Blockade of tissue factor eliminated thrombin generation, while inhibition of tissue factor pathway inhibitor significantly shortened LagT (p = 0.01) and TTP (P<0.0001), with a concomitant increase in endogenous thrombin potential.

**Conclusions/Significance:**

STBM triggered thrombin generation in normal plasma in a tissue factor dependent manner, indicating that TF activity is expressed by STBM. This is more pronounced in STBM shed from pre-eclampsia placentae. As more STBM are shed in pre-eclampsia these observations give insight into the disordered haemostasis observed in this condition.

## Introduction

Pre-eclampsia is a relatively common pregnancy-specific disorder affecting around 3% of pregnancies and is a major cause of fetal and maternal mortality and morbidity worldwide. It is characterized by hypertension, proteinuria, endothelial dysfunction and systemic activation of an inflammatory response [1]. During normal pregnancy, the placental syncytiotrophoblast releases microvesicles (STBM) and soluble inflammatory mediators in [2] to the maternal circulation [2], leading to a low-level physiological inflammatory response. In pre-eclampsia, there is increased release of STBM and other inflammatory factors that are thought to trigger the increased maternal inflammatory response characteristic of the disease [3]. Normal pregnancy is associated with a physiological increase in many procoagulant factors and inhibitors of fibrinolysis, such that fibrinolytic activity is reduced during pregnancy. In normal pregnancy, markers of *in vivo* thrombin generation (thrombin-antithrombin complexes [TAT], prothrombin fragment 1.2 [PF1.2] and D-dimer) are slightly increased as is the endogenous thrombin potential (ETP) [4].

The association between coagulation activation and pre-eclampsia has long been recognized and includes excessive platelet activation, increased fibrin degradation products and intervillous fibrin deposition in the placenta [5]. The shift in the haemostatic balance observed in normal pregnancy is exaggerated in pre-eclampsia. In practice, a spectrum of haemostatic changes are observed; from the subtle variation seen in in mild preeclampsia to disseminated intravascular coagulation. Tissue factor is a member of the cytokine receptor superfamily which is constitutively expressed by most non-vascular and perivascular cells and initiates the coagulation cascade following vascular injury [6]. It is essential for the development of embryonic blood vessels, migration and proliferation of vascular smooth muscle, and regulation of inflammation [7], [8]. The main physiological inhibitor of tissue factor in blood is tissue factor pathway inhibitor (TFPI), whereas tissue factor pathway inhibitor-2 (TFPI-2) is thought to be the main inhibitor of coagulation on the placental surface [9], although TFPI-2 acts primarily on factor Xa rather than tissue factor. It is thought that under normal circumstances cells in contact with blood do not express physiologically active TF [10]. The amount of tissue factor in the blood of normal individuals is controversial. Although circulating tissue factor has been reported in normal individuals at concentrations as high as 37pM [11], the consensus is that the level of circulating tissue factor in normal individuals is extremely low [12], [13], probably less than 20fM [14]. This is consistent with observations that sub-picomolar concentrations of tissue factor clot blood within a few minutes [10] and that tissue factor expressing pericardial microvesicles, but not normal plasma microvesicles, are thrombogenic *in vivo* [15]. Tissue factor bearing microvesicles are increased in several pathological states associated with thrombotic complications, e.g. sepsis, cancer and cardiovascular disease [16].

The presence of active tissue factor on the placental syncytiotrophoblast, which is in direct contact with the blood, is equally controversial. Although it has been reported to be present on membranes prepared by sonication of placental villi [17], choriocarcinoma cell lines [17], [18] and syncytiotrophoblasts differentiated *in vitro* from primary villous trophoblasts [19], histological studies have shown that it is present at high concentration in the decidua but absent from syncytiotrophoblasts [20]–[22]. However, more recently two groups [23], [24] have reported increased levels of tissue factor antigen and mRNA in the syncytiotrophoblast of placentae from women with pre-eclampsia.

The reasons for these conflicting reports may be the lack of standardization of methods for the measurement of tissue factor and poor specificity of the antibodies used [13]. It is now generally agreed that the measurement of tissue factor activity is more sensitive and specific than measurement of tissue factor antigen [10], [25]. Against this background, we studied the potential thrombogenicity of STBM shed from the maternal surface of the placenta as a model for the procoagulant state in pre-eclampsia.

## Results

There was no significant difference in maternal age, parity or body mass index between the normal and pre-eclamptic pregnancies at the time of booking. As would be expected, birth weight centile, gestational age and placental weight were all lower in pre-eclamptic pregnancies. The maternal platelet count fell an average of 73×10^9^/L in pre-eclamptic pregnancies but remained close to baseline, or above, in all except one normal pregnancy (Table 1).

**Table 1:** Patient characteristics.

Patient	Maternal age	BMI	Parity	Gestation (days)	Birth weight centile	Placental weight (g)	Platelet count ×10^9^/L	
							Booking	Pre-delivery
N1	28	42.5	1	273	37.3	NA	208	183
N2	29	24.4	1	273	25.7	NA	269	312
N3	26	17.6	1	272	20.4	563	208	169
N4	36	24.1	1	274	79.7	NA	221	243
N5	38	25.0	1	290	77.6	772	212	210
N6	33	NA	1	267	78.3	929	198	242
N7	34	21.5	0	294	49.6	613	210	135
N8	33	31.0	1	268	62	638	213	176
PE1	24	30.8	1	255	0.4	524	261	252
PE2	39	26.4	1	246	10.8	579	307	179
PE3	44	25.5	1	274	51.6	700	273	281
PE4	41	39.1	2	210	0.8	284	248	112
PE5	31	26.7	2	231	0.6	646	284	168
PE6	42	22.3	1	248	8.1	458	299	256
PE7	29	22.6	1	271	22.6	617	278	132
PE8	31	23.8	0	234	12.2	315	233	222

Platelet poor plasma (PPP) alone generated no thrombin upon recalcification. Endogenous thrombin potential (ETP) and peak thrombin formation were significantly increased by the addition of pre-eclampsia STBM compared to normal STBM, with concomitant reductions in median LagT and TTP (3.8 [IQR 2.4–6.8] v 8.3 [IQR 7.3–45.0] and 7.3 [IQR 4.6–12.4] v 15.8 [IQR 14.3–55.4] minutes respectively) (Fig. 1A). STBM from three of the normal pregnancy placentas generated little or no thrombin. By contrast, all pre-eclampsia STBM produced at least 300 nM of thrombin and reduced the LagT to less than 10 minutes. Preincubation with an inhibitory anti-tissue factor antibody eliminated all thrombin generation.

**Figure 1:** The effect of STBM on thrombin generation parameters of normal platelet poor plasma. (A) STBM were added to platelet poor plasma at a concentration 50 µg/mL. Following the addition of 4 µM phospholipid and 16 nM CaCl_2_, thrombin generation was monitored continuously. Endogenous thrombin potential (ETP), time to start of thrombin generation, peak thrombin generation and time to peak thrombin generation are shown for normal STBM and pre-eclampsia STBM (PET). (B) This was repeated after prior incubation with 25 µg/mL anti-TFPI and (C) 50 µg/mL anti-TFPI-2.

Blockade of TFPI resulted in all STBM preparations triggering a minimum ETP value of 680 nM when added to PPP, but was not sufficient to produce thrombin generation in PPP alone (Fig. 1B). Shorter LagT and TTP were observed with pre-eclampsia STBM than normal STBM. Preincubation with anti-TFPI-2 has no statistically significant effect of thrombin generation, although there was a trend towards increased ETP and peak (Fig. 1C).

The addition of recombinant tissue factor to PPP produced a dose response reduction in LagT (Fig. 2). These data indicate that the amount of active tissue factor present is approximately 0–100 pM/gram of protein on normal STBM and 40–800 pM/gram of protein for pre-eclampsia STBM (Table 2).

**Figure 2:** The effect of recombinant tissue factor on thrombin generation lag-time. Recombinant tissue factor was added to platelet poor plasma (final concentration 0.3–12pM). Following the addition of 4 µM phospholipid and 16 nM CaCl_2_, the mean lag time to start of thrombin generation was recorded. Error bars represent the standard deviation.

**Table 2:** Tissue factor content of syncytiotrophoblast microvesicles.

Sample	Lag time (s)	Tissue factor concentration (pg/g of protein)
N1	60.0	0
N2	7.8	51
N3	60.0	0
N4	40.7	7
N5	6.8	58
N6	7.5	54
N7	3.9	111
N8	8.7	47
PE1	9.7	43
PE2	4.0	106
PE3	6.3	63
PE4	3.6	123
PE5	8.5	48
PE6	2.6	225
PE7	1.6	812
PE8	2.0	401

N = normal STBM, PE + pre-eclampsia STBM.

It was notable that the only normal STBM sample (N7) estimated to contain in excess of 60 pM/gram of active tissue factor was from a patient whose platelet count had dropped by 75×10**^9^**/mL in the three weeks prior to delivery. Furthermore, two of the three pre-eclampsia STBM samples (PE1 and PE3) with less than 60 pM of tissue factor per gram of protein were obtained from patients with late onset pre-eclampsia who were not receiving anti-hypertensive therapy prior to delivery and whose platelet count remained stable throughout pregnancy.

## Discussion

Under normal circumstances, tissue factor is not expressed on endothelial cells and other cells in direct contact with the blood. Consequently, the presence, or otherwise, of tissue factor on the syncytiotrophoblast with the potential to initiate coagulation, in direct contact with maternal blood, has been controversial subject for many years. This controversy arises in part from poor methodological standardization which has led to conflicting reports. Although tissue factor antigen has been reported on the syncytiotrophoblast [17]–[24], the immunological methods used may also detect inactivated forms and alternatively spliced forms of the molecule which have no procoagulant activity [13].

We hypothesized that STBM shed during pre-eclamptic pregnancies into the maternal circulation contain increased levels of active tissue factor and that this could activate the coagulation system. Our study is unique in two respects: firstly, tissue factor activity rather than antigen was measured; and, secondly, this is the first time that tissue factor has been demonstrated on STBM rather than on the placental surface.

Our data confirm that negligible levels of active tissue factor exist in normal plasma, and that subpicomolar amounts of tissue factor can trigger coagulation [12]–[14]. The absence of thrombin generation in PPP demonstrates that contact factor inhibition by CTI in these experiments was complete. The absence of contact activation, the complete inhibition of thrombin generation by inhibitory tissue factor antibodies and the augmentation of thrombin generation by TFPI blockade demonstrate that the initiation of thrombin generation in these experiments was tissue factor specific.

STBM shed from the maternal surface of the placenta express significantly more active tissue factor in pre-eclampsia, as demonstrated by an increase in both the amount and rate of thrombin generation, with significantly shorter LagT and TTP compared to normals. Elimination of TFPI activity with inhibitory antibodies enhanced the sensitivity of the method, thus enabling the detection of active tissue factor in all STBM preparations. In contrast, blockade of TFPI-2 had minimal effect. This is consistent with the expression of low levels of tissue factor by syncytiotrophoblast in normal pregnancy. The increased levels of active tissue factor activity on STBM from pre-eclamptic pregnancies supports previous reports of upregulation of tissue factor on the syncytiotrophoblast during pre-eclampsia [23], [24]. However, in contrast to previous reports, we have demonstrated that this tissue factor is present in an active form capable of initiating coagulation in blood. Not only is there greater expression of tissue factor on pre-eclampsia STBM but significantly more are shed into the maternal circulation in pre-eclampsia, with estimates ranging from a 2–10 fold increase [26]–[30], which is consistent with reports of increased numbers of circulating STBM in the blood of women with pre-eclampsia [26], [31], [32] Together, these changes would be expected to comprise a substantial intravascular pro-thrombotic stimulus.

Two of the lowest pre-eclampsia STBM tissue factor activity levels were observed in women with mild late onset pre-eclampsia, who maintained a steady platelet count throughout pregnancy. By contrast, the women with severe early onset pre-eclampsia had high levels of STBM tissue factor activity. Of the eight STBM preparations obtained from normal pregnant women, only one had a significant elevation of tissue factor activity. This patient had a falling platelet count prior to delivery, which could be indicative of a developing procoagulant state . These data suggest that high tissue factor activity may precede overt disease and may be associated with more severe disease.

There have been many reports of increased circulating levels of tissue factor in pre-eclamptic women [29], [31], [33]–[35] but these measurements have all been made using immunological methods or poorly standardized functional assays, resulting in values several orders of magnitude higher than those obtained by specific functional assays. As subpicomolar quantities of tissue factor are now known to initiate clotting, it is highly unlikely that these measurements were detecting active tissue factor.

Given that tissue factor expression is generally in the order of pM, the small number of circulating STBM [26], [31], [36] and the rapid clearance of circulating microvesicles [37] and trophoblast debris [38], it is unlikely that tissue factor positive STBM persist in the circulation in sufficient numbers, or with sufficient antigen density, for accurate detection by flow cytometry. However, the shedding of tissue factor-bearing STBM into the maternal circulation would be expected to increase markers of *in vivo* thrombin generation and this is indeed the case [39]–[44].

While tissue factor is essential for placental and embryonic development, abberant expression is associated with poor pregnancy outcomes in mice [45]. Tissue factor has inflammatory functions, both dependent and independent of coagulation activation through the activation of protease-activated receptors (PARs) [7] on endothelial cells, platelets, neutrophils and monocytes. It has been reported that PAR-1 expression is increased on villous trophoblasts in pre-eclampsia [46] and that thrombin increases the release of soluble fms-like tryrosine kinase (sFLT-1), a potent anti-angiogenic factor and a key player in pre-eclampsia [47] suggesting a role for tissue factor and thrombin in the pathogenesis of pre-eclampsia.

This study had some limitations.

Placental tissue factor is heavily glycosylated and is reported to be 5-fold more active than recombinant tissue factor [48]. Consequently, we may have overestimated STBM tissue factor expression as our calibration curve was performed using recombinant tissue factor.

It was not possible to perfuse all the placentae obtained due to excessive placental infarction or mechanical damage. Furthermore the lobules selected for perfusion were those which were not obviously infarcted. Consequently the samples collected may have been biased towards less severe forms of pre-eclampsia. Due to logistical issues, only those cases delivered by elective caesarean section could be included which would also have excluded inclusion of fulminating disease with emergency delivery.

We cannot discount the possibility that tissue factor was produced *ex vivo* during the perfusion. However, this would not explain the difference in tissue factor activity between normal and pre-eclampsia placentae.

Blood samples were not obtained from the women prior to delivery, so it was not possible to relate STBM tissue factor levels with *in vivo* markers of thrombin generation.

In conclusion, we have shown that the placenta releases tissue factor bearing microvesicles from the maternal face of the placenta and tissue factor activity is increased in STBM released during pre-eclampsia. The low level shedding of active tissue factor into the maternal circulation via STBM may be responsible for the physiologically important procoagulant state in normal pregnancy. It is probable that the increased rate of STBM shedding combined with higher tissue factor expression may contribute to maternal inflammation and disordered hemostasis observed in pre-eclampsia.

## Materials and Methods

### Patient details

Placentae were obtained at caesarean section, without labour, from healthy pregnant women or women with pre-eclampsia. Women with pre-existing renal disease, previous surgery, insulin-dependent diabetes or asthma requiring steroidal treatment were excluded. Pre-eclampsia was diagnosed by new hypertension after the 20^th^ week of pregnancy (diastolic blood pressure ≥90 mmHg on at least two occasions) and new proteinuria (2+ protein on dipstick testing on 2 occasions; ≥500 mg/24 hour; or ≥50 mg/ml protein/creatinine ratio) in the absence of urinary tract infection. Inclusion criteria for normal pregnancy were: singleton pregnancy, normal obstetric history; diastolic <90 mmHg and systolic blood pressure <140 mmHg; and no significant proteinuria (<1+) and congenitally normal livebirth at term. The study was approved by the Mid and South Buckinghamshire Research Ethics Committee and all participants gave written informed consent.

### Reagents

Corn trypsin inhibitor (CTI) was purchased from Cambridge Bioscience (Cambridge, UK). The antibodies used were: NDOG2 an in-house anti-syncytiotrophoblast antibody which recognizes placental alkaline phosphatase [27]; polyclonal rabbit anti-human tissue factor antibody, polyclonal rabbit anti-human TFPI (American Diagnostica Inc. CT) and monoclonal anti-human TFPI-2 (R&D Systems, Abingdon, UK). Fc receptor blocker was obtained from Miltenyi Biotec, Bergisch Gladbach, Germany. Thrombin generation was measured using MP Reagent (containing 4 µM phospholipid, final concentration), start reagent (FluCa™; containing 1/40 volume fluorogenic substrate, 16.7 nM calcium chloride, Hepes, pH 7.35) and Thrombin Calibrator (all Diagnostica Stago, Asnières sur Seine, France).

### Plasma preparation

The substrate plasma was prepared from blood collected from a single normal fasting donor using a 19 G needle with minimal suction and a light tourniquet into 0.106 mmol trisodium citrate containing corn trypsin inhibitor (final concentration 20 µg/mL). Platelet poor plasma (PPP) was prepared by double centrifugation at 2500 **g** for 15 minutes with supernatant separation, and frozen at −80°C until required.

### Preparation of syncytiotrophoblast vesicles (STBM)

STBM were prepared using a dual placental perfusion system [32]. Briefly, placentae obtained at caesarean section, without labour were processed immediately. The whole placenta was laid inside a Perspex water jacket maintained at 37°C. The fetal circulation of a single lobule, not visibly infarcted, was perfused with 0.1 µm filtered modified M-199 tissue culture medium, containing 0.8% Dextran 20, 0.5% BSA, 5000 U/L sodium heparin and 100,000 IU streptokinase at a rate of 5 mL/min. The maternal side was perfused with modified M-199 tissue culture medium containing 0.5% BSA and 5000 U/L sodium heparin at a controlled rate of 20 ml/min and oxygenated with 95% O2, 5%CO2. To equilibrate the system, the lobule was initially perfused for 20 min and the effluent of the maternal and fetal circuits was discarded. After this time the maternal circuit was closed containing 600 ml of fresh perfusion medium. The volume of fetal effluent was measured every 2 min and the oxygen concentration of the maternal side perfusate monitored continuously to ensure stability. Pressure monitors were used on both the maternal and fetal sides of the placenta to ensure no significant deviations from baseline during the experimental period. After 3 hr, the maternal perfusate was centrifuged at 600 ***g*** for 10 min to remove cellular debris. The remaining supernatant was ultracentrifuged at 150,000 ***g*** to pellet the STBM. The resultant pellets were pooled and washed in phosphate buffered saline (PBS) and then resuspended in PBS to a final total protein concentration (BCA protein assay kit) of 5 mg/ml and stored in aliquots at −80°C until use. Of the 10 normal and 10 pre-eclampsia placentas collected for this study, it was not possible to perfuse three pre-eclampsia placentas and two normal placentas due to infarction or mechanical damage. The placental origin of the STBM was verified by flow cytometry using NDOG2, a trophoblast specific monoclonal antibody which recognises placental alkaline phosphatase [49]. All STBM samples were blocked with Fc receptor blocker for 10 min at 4°C before the addition of NDOG2-FITC or IgG_1_ FITC isotype control. Flow cytometry analysis was performed on a BD LSRII flow cytometer (BD Biosciences), and data were analyzed by FACSDIVA software. There was no significant difference in the percentage of STBM which stained with the NDOG2 antibody between the normal and pre-eclampsia STBM (median 91.7% v 85.3%; P = NS).

### Thrombin generation

Perfused STBM were diluted to 500 ng/mL and pre-incubated with PBS, anti-TFPI, anti-TFPI-2 or anti-tissue factor. This suspension was then added to PPP (final concentration; STBM 50 µg/mL; anti-TFPI 25 µg/mL; anti-TFPI-2 50 µg/mL and anti-TF 20 µg/mL). Calibrated automated thrombin generation was measured according to the method of Hemker et al. [50] with the addition of 20 µg/mL CTI to prevent contact factor activation [51]. Briefly, 80 µL of sample per well were added to a 96 well plate followed by 20 µL of MP Reagent or 20 µL Thrombin Calibrator. After incubation at 37°C for 20 minutes 20 µL start reagent were added. Fluorescence intensity was measured continuously for 60 minutes using a fluorescent plate reader (Fluoroskan Ascent FL, Thermo Electron Corporation, Helsinki, Finland) equipped with a 390/460 nm filter set. The fluorescent signal was converted into thrombin concentration using the internal thrombin calibrator and dedicated software (Thrombinoscope bv, Maastricht, Netherlands). All samples with and without calibrator were tested in duplicate wells. The endogenous thrombin potential (ETP; i.e., the area under the curve) peak thrombin generation (peak), lag time to start of thrombin generation (LagT), time to peak thrombin generation (TTP), and were recorded. If no thrombin generation was observed, the LagT and TTP were recorded as 60 minutes. In CTI-treated plasma, and in the presence of phospholipid, LagT is largely dependent on tissue factor activity [12]. In order to estimate tissue factor concentration, recombinant human tissue factor was added to plasma (final dilutions of 0.3–12.0 pM) prior to measurement of thrombin generation and tissue factor concentration was plotted against LagT as previously described [12].

### Statistics

Statistical analyses were performed using Graphpad Prism software. Nonparametric statistics were used unless otherwise stated. The statistical significance of differences between groups was determined by the Mann Witney U test. *P* values <0.05 were considered significant.
